This article has been retracted.

# Decreased long intergenic noncoding RNA P7 predicts unfavorable prognosis and promotes tumor proliferation via the modulation of the STAT1-MAPK pathway in hepatocellular carcinoma

**DOI:** 10.18632/oncotarget.23282

**Published:** 2017-12-08

**Authors:** Sijie Cheng, Tieling Li, Cheng Wang, Keyu Wang, Chengcai Lai, Jin Yan, Hongxia Fan, Fang Sun, Zhaohai Wang, Peirui Zhang, Linxiang Yu, Zhixian Hong, Guanglin Lei, Baijun Sun, Yuan Gao, Zhaohui Xiao, Xu Ji, Ruilan Wang, Jianzhong Wu, Xiliang Wang, Shaogeng Zhang, Penghui Yang

**Affiliations:** ^1^ Beijing 302 Hospital, Beijing, 100039, China; ^2^ Chinese PLA General Hospital, Beijing, 100853, China; ^3^ State Key Laboratory of Pathogens and Biosecurity, Beijing Institute of Microbiology and Epidemiology, Beijing, 100071, China

**Keywords:** HCC, long noncoding RNA, lincRNA P7

## Abstract

Hepatocellular carcinoma (HCC) is the most common neoplasm and is a leading cause of cancer-related death. Despite advances in the diagnosis and management of HCC, its prognosis remain unfavorable. Accumulating evidence has shown that long intergenic noncoding RNAs (lincRNAs) play central roles in the development of HCC. In this study, we identified a long intergenic noncoding RNA referred to as lincRNA P7 in HCC and explored its clinical significance and biological functions in HCC. The expression level of lincRNA P7 was significantly aberrantly deceased in HCC cancer tissues and cells lines. Gain- and loss-of-function experiments revealed that overexpression of lincRNA P7 significantly inhibited the proliferation of HCC-derived cancer cells, whereas lincRNA P7 knockdown promoted cell growth. Mechanistically, lincRNA P7 blocked Erk1/2 signaling and repressed activation of the STAT1 pathway. In nude mouse models, we show that overexpression of lincRNA P7 effectively repressed HCC xenograft tumor growth *in vivo*. Moreover, a clinical investigation demonstrated that down-regulated lincRNA P7 expression correlated with liver cirrhosis, Hepatitis B virus (HBV) infection, clinical stage of the tumor and recurrence. A Kaplan-Meier survival analysis showed that the expression of lincRNA P7 was significantly related to overall survival (*P* = 0.003) and recurrence-free survival (*P* = 0.031). Collectively, our findings suggested that the down-regulation of lincRNA P7 predicts poor clinical outcomes for HCC patients and might be a powerful candidate prognostic biomarker and target in HCC.

## INTRODUCTION

Liver cancer is a major health problem [1] and is currently the second leading cause of cancer-related death worldwide [2]. Among all primary liver cancers, hepatocellular carcinoma (HCC) is the most common neoplasm, as it accounts for approximately 90% of cases [3]. Liver cirrhosis, hepatitis B virus (HBV) infection, hepatitis C virus (HCV) infection, alcohol abuse, metabolic syndrome and other risk factors are well defined factors that contribute to the development of HCC. Other co-factors such as tobacco inhalation and uptake of aflatoxin B1 are also recognized contributors to the development of HCC [4]. Recent studies have demonstrated that adeno-associated virus 2 (AAV2) infection is a novel contributor to the disease [5]. Some main pathways with components that are frequently mutated in HCC such as the telomere maintenance pathway, the cell cycle pathway, WNT-β-catenin, and epigenetic and chromatin remodeling pathways have been well described [6–12]. Despite progress in the diagnosis, prevention and treatment of HCC, its prognosis remains unfavorable. Even after curative therapy, the median survival rate remains lower than 50% for 5 years [13–15].

LncRNAs are noncoding transcripts that surpass 200 nt in length and have been described as the largest subclass of the noncoding transcriptome in humans [16]. Most lncRNAs are transcribed by RNA polymerase II, and they are thus capped and polyadenylated at their 5′ and 3′ ends, respectively. LncRNAs generally do not encode proteins, but many of them are able to code for oligopeptides. With the development of microarrays and high-throughput sequencing technologies, the recent growing number of cancer transcriptomes has indeed revealed thousands of long noncoding RNAs (lncRNAs) whose aberrant expression is associated with different cancer types [17–19] including HCC. Several lncRNAs such as HULC [20], CCAT1 [21], PXN-AS1 [22], TSLNC8 [23], and ATB [24], among others, have been shown to be dysregulated and to play crucial roles in HCC progression. However, the expression, roles and functional mechanisms of lncRNAs in HCC are still largely unknown.

In this study, we identify and explore the expression levels of the lincRNA P7 in HCC tissues and its relationship with the clinic-pathological features of HCC. In addition, the roles, underlying functional mechanisms and clinical significance of lincRNA P7 in the progression of HCC were also investigated.

## RESULTS

### lincRNA P7 is preferentially down-regulated in HCC cancer tissues

To identify the deregulated lncRNA profiles in HCC patients, we performed a lncRNA microassay analysis in a set of cancer tissues and paired non-tumor tissues derived from 5 HCC patients. Interestingly, we identified 503 lncRNAs (128 up-regulated, 375 down-regulated) along with 1300 mRNAs (648 up-regulated, 652 down-regulated) from a total of 9759 lncRNAs and 18,627 mRNAs based on dysregulated fold changes > 2 (Supplementary Figure 1, Supplementary Table 1). We then performed a lncRNA and mRNA co-expression analysis and found that the expression levels of 7 lncRNAs were significantly correlated with their corresponding 25 mRNAs (Figure 1A and Supplementary Table 1). Moreover, we analyzed the GO and PATHWAY results and found that the ko05200 Pathway in cancer and the ko04020 MAPK pathway were the two primary pathways with alterations in HCC (Figure 1B, Supplementary Table 1). Then, we verified the expression level of 7 of the above lncRNAs in the normal human liver cell line LO2 and in the HCC cell lines HepG2, Huh7 and SMMC-7721. We found 4 altered lncRNAs, which was consistent with the microarray results (Supplementary Figure 2A); the lncRNAs XR15898, lncRNA XR429178.1, linc-TET2-5 and lincRNA P7 exhibited remarkable fold changes (> 10-fold) (Supplementary Table 1). We next re-verified their expression in 18 paired adjacent noncancerous hepatic tissues, and the results showed that lincRNA P7 was the most differentially expressed among these lncRNAs (Supplementary Figure 2B). The lincRNA P7 is an annotated lincRNA 581 nt in length (Supplementary Figure 1C) that is located on chromosome 7 in humans and on the gene RP11-30J20.1 (ENST00000520060.1). Therefore, we focused on the uncharacterized lncRNA and lincRNA P7 in subsequent studies.

**Figure 1:** LincRNA P7 is preferentially down-regulated in HCC tissues (**A**) Hierarchical clustering of the expression level of the 7 most variable lncRNAs was significantly correlated with their corresponding 25 mRNAs. LincRNA P7 is marked in red. Expression values are indicated as high (red) or low (green). (**B**) PATHWAY analysis of the microarray results.

### lincRNA P7 is significantly decreased in human HCC tissues and cell lines

To explore the role of the lincRNA P7 in HCC progression, we first examined the lincRNA P7 expression level in 108 pairs of HCC tissues and adjacent non-tumor tissue specimens by qRT-PCR. As shown in Figure 2, lincRNA P7 levels were significantly decreased in HCC tissues compared with matched adjacent non-tumor tissues (*P* < 0.001, Figure 2A, 2B). LincRNA P7 expression was also examined in three human HCC cell lines (SMMC-7721, HepG2 and Huh7) and in the normal liver cell line LO2. This experiment revealed down-regulated lincRNA P7 expression in all three HCC cell lines compared with LO2 cells (*P* < 0.05, Figure 2C). Moreover, receiver operating characteristic (ROC) curves were used to evaluate the sensitivity and specificity of lincRNA P7 expression in order to discriminate between the tumor and control samples. Notably, lincRNA P7 exhibited predictive behavior with an area under the curve (AUC, represents discrimination accuracy) of 0.743 (Figure 2D), which suggests that the level of lincRNA P7 demonstrated adequate sensitivity and specificity to discriminate between HCC tissues and adjacent non-tumor tissues. Additionally, a nucleocytoplasmic separation experiment showed that lincRNA P7 was predominately located in the cytoplasm (Figure 2E). Taken together, these data indicated that lincRNA P7 may be clinically significant in the diagnosis of HCC and may play a critical role in HCC progression.

**Figure 2:** LincRNA P7 expression levels in HCC tissues and cells (**A**) Relative expression levels of lincRNA P7 in tumor tissues compared with adjacent normal tissues (*n* = 108). LincRNA P7 expression was evaluated by qRT-PCR and normalized to GAPDH expression. (**B**) Positive values for lincRNA P7 expression indicate a higher level of lncRNA expression in tumor tissue compared with nontumor tissue, while negative values indicate a lower level of lincRNA P7 expression in tumor tissue compared with adjacent tissue. (**C**) The level of lincRNA P7 expression was lower in HCC cell lines than in the normal liver cell line LO2 (^***^p < 0.001). (**D**) The area under the receiver operating characteristic (ROC) curve for the prediction of HCC based on lincRNA P7 expression, which used the corresponding adjacent normal tissues as controls. (**E**) qRT-PCR analysis of lincRNA P7 in the subcellular fractions of SMMC 7721 and Huh7 cells. U6 and β-actin served as nuclear and cytoplasmic markers, respectively (*n* = 3).

### Enforced expression of lincRNA P7 suppresses HCC cell proliferation *in vitro*

To investigate the biological functions of lincRNA P7 in HCC, we stably enhanced lincRNA P7 expression via the transfection of the HCC cell lines SMMC7721 and Huh7 with the lincRNA P7 expression vector pcDNA3.1- lincRNA P7. Empty vector was used as a negative control (Figure 3A). Cell-counting kit 8 (CCK8) assays showed that overexpression of lincRNA P7 in the HCC cell lines SMMC7721 and Huh7 significantly reduced the cell proliferation ability of these cells. SiRNA-2 in SMMC7721 and siRNA-1 in Huh7 had no significant effect on HCC cell proliferation in comparison with the control (Figure 3B). Colony formation assays also indicated that the SMMC7721 and Huh7 cells transfected with lincRNA P7 formed significantly fewer colonies than control SMMC7721 and Huh7 cells (Figure 3C). Moreover, we inhibited lincRNA P7 expression by transfection of SMMC7721 and Huh7 cells with lincRNA P7-specific siRNA. As demonstrated by CCK-8 assays, the repression of lincRNA P7 significantly increased the proliferation of SMMC7721 and Huh7 cells. Colony formation assays indicated that lincRNA P7 repressed colony formation in SMMC7721 and Huh7 cells, as they formed fewer colonies than control SMMC7721 and Huh7 cells. Next, flow cytometric analysis was performed to examine whether the effects of lincRNA P7 on proliferation of HCC cells by altering apoptosis or cell cycle progression. The results showed that lincRNA P7 couldn't affect apoptosis and cell cycle of these cells (Supplementary Figure 3). Overall, these results suggested that lincRNA P7 has a crucial function in the regulation of HCC cell proliferation.

**Figure 3:** LincRNA P7 inhibited the proliferation of HCC cells *in vitro* (**A**) LincRNA P7 overexpression and knockdown in HCC cells lines. The expression level of lincRNA P7 was robustly enhanced or reduced when the cell lines were treated with pcDNA3.1-LincRNA P7 or with two siRNAs that target lincRNA P7, respectively. Empty vector and the siRNA control were used as the negative controls. (**B**) MTT assays were used to determine the cell viability of si-LincRNA P7- and pCDNA- LincRNA P7-transfected SMMC7721 and Huh7 cells. Cell number was determined every 24 h for a total of 96 h using CCK-8 assays. The results are shown as the means ± s.e.m. from three independent experiments. ^*^P < 0.05, compared with the control by two-sided *t*-test. (**C**) Colony-forming assay was conducted to determine the effect of lincRNA P7 on the proliferation in SMMC7721 and Huh7 cells. (**D**) LincRNA P7 regulates the STAT1 and MAPK signaling pathway. Immunoblot analysis showed that the phosphorylation of STAT1 (pSTAT1) and Erk1/2 (pErk1/2) was significantly repressed in lincRNA P7-overexpressing SMMC7721 and Huh7 cells. In contrast, the phosphorylation of these proteins was rescued in si-lincRNA P7-transfected SMMC7721 and Huh7 cells.

Based on the above pathway analysis, we presumed that lincRNA P7 might affect HCC cell proliferation via the MAPK pathway. To explore whether the effects of lincRNA P7 on HCC cells are associated with this pathway, we evaluated the activity of lincRNA P7 on a component of this pathway (Erk protein). As shown in Figure 3D, phosphorylation of Erk1/2 was significantly suppressed after the transfection of SMMC-7721 and Huh7 cells with pcDNA3.1- lincRNA P7. The total amount of Erk1 and Erk2 (Erk1/2) protein expression was not significantly different in cells that overexpressed lincRNA P7; however, the level of phosphorylated Erk1/2 was remarkably decreased in cells that overexpressed lincRNA P7 relative to control cells (Figure 3D).

Signal transducer and activator of transcription 1 (STAT1), which is known as an upstream component of the MAPK pathway, has a critical role in the regulation of cell proliferation. To explore whether the effects of lincRNA P7 on HCC cells are related to STAT1 protein, we also assessed the STAT1 levels in cells with altered lincRNA P7 expression and found that overexpression of lincRNA P7 decreased the levels of phosphorylated STAT1, whereas the knockdown of lincRNA P7 showed the opposite effect to increase the levels of phosphorylated STAT1 (Figure 3D). Then, to address whether blockade of the Erk1/2 and STAT1 signaling using specific inhibitors would affect cell proliferation of HCC cells, SCH772984 [25] and Fludarabine [26] were used to inhibit Erk1/2 and STAT1, respectively. CCK-8 and colony formation assays were performed to determine the effects of lincRNA P7 on HCC cell growth in presence of SCH772984 or Fludarabine. The results showed that SCH772984 or Fludarabine could inhibit the SMMC7721 cells proliferation and could abolish the surppression of HCC cells proliferation induced by lincRNA P7 (Supplementary Figure 4). These findings suggested that the effects of lincRNA P7 are associated with the STAT1-MAPK pathway. We further analyzed the correlations between lincRNA P7 levels and the mRNA levels of the STAT1 and Erk1/2 genes in 60 clinical HCC tissue samples, and found no significant correlations between lincRNA P7 and the mRNA levels of Erk1/2 and STAT1 (Supplementary Figure 5). These results suggested that lincRNA P7 might suppress HCC proliferation via the regulation of the STAT1-MAPK signaling pathway in HCC cells.

### Enforced expression of lincRNA P7 represses HCC xenograft tumor growth *in vivo*

Subsequently, we explored whether low levels of lincRNA P7 expression could suppress tumor growth *in vivo*. SMMC7721 cells that stably overexpressed lincRNA P7 or empty vector were inoculated into nude mice. As demonstrated in Figure 4, we found that the growth rate of the tumors in the pcDNA3.1- lincRNA P7 group was slower than that in the empty vector group. Five weeks after injection, tumors dissected from the mice in the pcDNA3.1- lincRNA P7 group were significantly smaller than those of their control counterparts. The higher expression levels of lincRNA P7 were observed from tumor in the pcDNA3.1-lincRNA P7 group. Meanwhile, western blotting results showed that expression levels of phospho-Erk1/2 and phospho-STAT1 decreased in the tumors from mice in the pcDNA3.1-lincRNA P7 group compared with empty vector group. Additionally, the differences in weight of the nude mice in the two groups were not significantly different (Supplementary Figure 6). In contrast, the tumor volumes and weights were markedly lower in the pcDNA3.1- lincRNA P7 group than in the empty vector group, which demonstrated that lincRNA P7 represses the growth of HCC xenograft tumors *in vivo*.

**Figure 4:** Effects of lincRNA P7 down-regulation on tumor growth in a nude mouse model (**A, B**) SMMC7721 cells (5 × 10^6^) that stably expressed lincRNA P7 were inoculated into nude mice, and the effect of lincRNA P7 on HCC tumor growth was examined every 3 days for 42 days (6 weeks) (*n* = 6). The results show that lincRNA P7 significantly increased the proliferation of HCC tumor cells compared with the control lentiviral vector in nude mice. ^***^P < 0.001 (**C**) Tumor weight in each of the two groups is shown. The results are presented as the means ± s.d. for six mice in each group. ^*^P < 0.05, compared with control cells by two-sided *t*-test. (**D**) Effect of lincRNA P7 on HCC growth was described by tumor/body weight ratio in the two groups. Data are shown as the mean ± s.d. ^**^P < 0.01. (**E**) The expression levels of lincRNA P7 were determined by qRT-PCR in the xenograft tumors. (**F**) The expression levels of the phospho-Erk1/2 and phospho-STAT1 were determined by Western Blotting in the xenograft tumors.

### Relationship among lincRNA P7 expression, clinical parameters and patient prognosis

To determine whether lincRNA P7 expression in HCC tissues determines the clinical progression and outcome of HCC patients, we divided the 108 HCC patients into a high lincRNA P7 expression group (above average expression, *n* = 54) and a low lincRNA P7 expression group (below average expression, *n* = 54). As shown in Supplementary Table 1, lincRNA P7 expression was either closely associated with liver cirrhosis (*p* < 0.001), HBV infection (*p* < 0.001), clinical tumor stage (*p* < 0.05) and recurrence (*p* < 0.05). In contrast, no obvious differences were observed in age, number of tumors, AFP level, and portal vein tumor thrombus (PVTT), among other parameters (*p* > 0.05).

We further examined whether the lincRNA P7 expression level was correlated with the outcome of HCC patients. We next categorized patients into 2 cohorts, as follows: patients with lincRNA P7 expression values below the 50th percentile were classified as having lower lincRNA P7 levels (*n* = 54); patients with lincRNA P7 expression values above the 50th percentile were classified as having higher lincRNA P7 levels (*n* = 54). A Kaplan-Meier analysis of 108 patients with HCC revealed that a lower lincRNA P7 expression level in HCC tissues was significantly correlated with a reduction in overall survival (*p* = 0.003; Figure 5A) and recurrence-free survival (*p* = 0.031; Figure 5B). These data revealed that lincRNA P7 may play a vital role in the progression and outcomes of HCC.

**Figure 5:** Aberrant expression of lincRNA-P7 and the overall survival and recurrence-free survival rates Kaplan-Meier analyses of the correlations between the lincRNA P7 expression level and overall survival (**A**) and recurrence-free survival (**B**) of 108 patients with HCC. The median expression level was used as the cutoff. Patients with lincRNA P7 expression values below the 50th percentile were classified as having lower lincRNA P7 levels. Patients with lincRNA P7 expression value above the 50th percentile were classified as having higher lincRNA P7 levels.

## DISCUSSION

With advancements in deep sequencing technology, numerous lncRNAs have been found to be differentially expressed in cancers. Among these aberrant lncRNAs, several have been verified to be critical regulators of biological processes, including cell proliferation, in cancer. Herein, our microassay data have revealed that lincRNA P7 is dysregulated. This lncRNA acts as a tumor suppressor in several types of cancer and may help regulate the pathogenesis of HCC.

In this study, we identified the differential expression of lincRNA P7 between HCC tissues and matched adjacent non-tumor liver tissues using a microarray analysis. Our results showed that lincRNA P7 was down-regulated in HCC tissues compared with matched non-tumor liver tissues. The area under the ROC curve of lincRNA P7 was 0.743, which shows its specificity and sensitivity in the diagnosis of HCC. We also identified the function of lincRNA P7 in HCC cells through the application of gain-of-function and loss-of-function approaches. Overexpression of lincRNA P7 inhibits the proliferation of HCC cells, while the knockdown of lincRNA P7 promotes the proliferation of HCC cells. Furthermore, our *in vivo* experiment revealed that lincRNA P7 suppresses tumor growth in nude mice. Clinically, down-regulated lincRNA P7 is closely correlated with liver cirrhosis, HBV infection, clinical tumor stage and recurrence. Lower lincRNA P7 expression in HCC tissues indicated poor overall survival and recurrence-free survival of HCC patients. Therefore, our results showed that lincRNA P7 may play an important role in the development and progression of HCC.

Several studies have shown that MAPK signaling is a vital pathway that participates in cell proliferation [27, 28]. Blockade of the MAPK pathway has been considered useful in cancer treatment. Based on our findings, we speculated that lincRNA P7 might regulate targeted protein expression partly through inactivation of the MAPK pathway. Further studies are needed in order to gain insight into the mechanisms by which lincRNA P7 regulates the MAPK signaling pathway.

Previous studies have shown that liver cirrhosis is a predictor of recurrence of HCC and is an independent risk factor for HCC recurrence, and patients with liver cirrhosis tend to express different levels lncRNAs [29]. Clinical patients with liver cirrhosis are usually resistant to direct-acting antiviral (DAA) drugs, which results in a higher probability of tumorigenesis once these patients are infected with the HBV or HCV virus. HCC frequently develops during the advanced stage of fibrosis stage, and thus the eradication of HBV or HCV infection has been a promising prophylactic therapy for the prevention of the occurrence of liver fibrosis and HCC [30]. Several lncRNAs have been confirmed to participate in HCC progression, but few studies have reported the function of lncRNA in cirrhosis. On the contrary, the lncRNA HULC was found to be up-regulated in plasma samples from patients with HBV-related cirrhosis [20, 31]. We observed that low lincRNA P7 expression in patients is associated with cirrhosis, which is consistent with previous findings and suggests that some specific lncRNA expression profiles may be altered in HCC patients with cirrhosis. Of course, the effect of lincRNA P7 in HCC and potential lincRNA P7 targets need to be further investigated.

In conclusion, our results demonstrated for the first time that lincRNA P7 levels were significantly decreased in HCC tissues, which promoted tumor cell proliferation via the modulation of the STAT1-MAPK pathway *in vitro*. In addition, dysregulation of lincRNA P7 was positively correlated with liver cirrhosis, HBV infection, clinical tumor stage and recurrence in HCC patients. HCC patients with low levels of lincRNA P7 expression exhibited a significantly shorter OS and RFS than patients with higher expression of lincRNA P7. These findings demonstrate that lincRNA P7 is an important marker for the prediction of prognosis and may have potential as a diagnostic and therapeutic target in HCC.

## MATERIALS AND METHODS

### Clinical samples

Data from 108 consecutive patients (88 males and 20 females) who underwent surgery for HCC at Beijing 302 Hospital between August 2013 and April 2017 were accessed from the records of the hospital's Department of Hepatobiliary Surgery. Tumor tissues and adjacent non-tumor tissue specimens were collected from the patients after informed consent was obtained, which was in accordance with the institutional guidelines of the hospital's Ethics Committee. Resected tumor tissue and adjacent normal tissue specimens were immediately snap-frozen in liquid nitrogen and stored in a tissue bank until use.

### Cell lines and cell cultures

The human cell lines used in this study were obtained from the Experimental Guarantee Center of Beijing 302 Hospital (Beijing, China), and included the liver cancer cell lines HepG2, Huh7 and SMMC-7721 and the normal human liver cell line LO2. All of the cell lines were maintained in an atmosphere of 5% CO_2_ and were grown in DMEM medium (Thermo, Beijing, China) supplemented with 10% fetal bovine serum (Gibco, Beijing, China).

### RNA extraction and real-time PCR

Total RNA from frozen HCC tissues and adjacent non-tumor tissue samples were extracted using TRIzol reagent (Invitrogen Life Technologies, Carlsbad, CA, USA) according to the manufacturer's protocol. RNA integrity was evaluated using a NanoDrop ND-1000 spectrophotometer (NanoDrop Products, Wilmington, DE, USA), and cDNAs were synthesized from 50 ng total RNA from each sample. LincRNA P7 expression levels were quantified by qRT-PCR performed in an ABI7500 system (Applied Biosystems, Foster City, CA, USA) using Maxima SYBR Green qRT-PCR master mix (Thermo Fisher Scientific, Waltham, MA, USA) according to the manufacturers' protocols. GAPDH expression was monitored as the endogenous control, and all samples were normalized to human GAPDH. All reactions were run in triplicate, and the lincRNA P7-specific primers used were designed and synthesized by Sangon Biotech (Sangon, Shanghai, China). Their sequences were as follows: qRT-PCR primers of lincRNA P7 forward: 5′- TGTGAACC AGGTTTGCTGGA -3′, reverse: 5′- CTCAACCATGCC GACGAGAA -3′; GAPDH forward: 5′-CAGCCTCAAGAT CATCAGCA-3′ reverse: 5′-TGTGGTCATGAGTCCTT CCA-3′. The amplification profile was 95°C for 5 min, followed by 40 cycles of denaturation at 95°C for 15 s, and annealing at 60°C for 30 s. The median of triplicate reactions was used to calculate the relative lncRNA expression (ΔCt = Ct median lncRNA - Ct median GAPDH). Fold changes in expression were calculated using the 2^−ΔΔCt^ method.

### Vector construction

The lincRNA P7 overexpression vector was constructed in our laboratory and was sub-cloned into the BamHI and EcoRI sites of the pcDNA3.1 (+) vector, which yielded pcDNA3.1-lincRNA P7. The primers used in vector construction were as follows: forward: 5′- AGCTG AGGGAGCCGGCT -3′, reverse: 5′- ATTAATGAGA GAA TTATGGTAT -3′. Two siRNAs were synthesized by RIBOBIO CO., LTD (Guangzhou, China). The sequence of siRNA-lincRNA P7-1 was: 3′- dTdT GGCUCAGU CUUUGAUCAAA -5′; the sequence of siRNA-lincRNA P7-2 was: 3′- dTdT CCUGUAGUAAACUACUCAA -5′. The number of the siRNA negative control purchased from RIBOBIO is siN05815122147, but its specific sequence is not shown. The SMMC7721 cell line stably transfected with a lentiviral vector containing lincRNA P7 was constructed by Hanbio Biotechnology Co., Ltd. (Shanghai, China).

### Nucleocytoplasmic separation experiment

The nucleocytoplasmic separation experiment used Ambion Life Technologies PARIS^TM^ Kit, Protein and RNA Isolation system (Lithuania). This experiment was performed according to the instructions provided by the kit.

### Cell proliferation assay

Cell proliferation was assayed by Cell Counting Kit-8 (Dojindo Laboratories, Kumamoto, Japan) according to the manufacturer's instructions. Huh7 or SMMC7721 cells were plated in 12-well plates (5 × 10^5^ cells/well), and for the cells that overexpressed lincRNA P7, the number of cells per well was measured by the absorbance (450 nm) of reduced WST-8 (2-(2-methoxy-4- nitrophenyl)-3-(4-nitrophenyl)-5-(2,4-isulfophenyl)-2H-tetrazolium, monosodium salt) at the indicated time points. To block Erk1/2 and STAT1 signaling, SMMC7721 cells were treated with SCH772984 (4 nM) and Fludarabine (5 μM) for 6 h, respectively. After a certain time in culture, cell viability was measured using CCK-8 assays.

### Colony formation assay

Two hundred cells were plated into 6-well plates and incubated in DMEM with 10% FBS at 37°C. Seven days later, the cells were fixed and stained with 0.1% crystal violet. The number of colonies, defined as > 50 cells/colony, were then counted. To block Erk1/2 and STAT1 signaling, SMMC7721 cells were treated with SCH772984 (4 nM) and Fludarabine (5 μM) for 96 h, respectively. The cells were fixed and stained with 0.1% crystal violet after fortnight.

### *In vivo* experiments

The nude BALB/C mice (4-weeks-old) were purchased from the Chinese Academy of Military Medical Science (Beijing, China) and were maintained in a specific pathogen-free facility. SMMC7721 cells (2 × 10^6^) that stably overexpressed lincRNA P7 or empty vector were subcutaneously injected into the flanks of nude mice (*n* = 6 /group). Tumor growth was monitored by tumor weight, which was calculated at the indicated time points. Tumor volumes were calculated using the following formula: tumor volume (mm^3^) = length × width^2^ × 0.5.

### Statistical analysis

All data were expressed as the mean ± SD. For comparisons, Student's *t*-test or Chi-squared test were performed as indicated. Kaplan-Meier analyses were performed to determine the correlations between the lincRNA P7 expression level and the overall survival rate (OS) or recurrence-free survival (RFS). All statistical analyses were performed using the SPSS 18.0 software package (Chicago, IL, USA). *P* values < 0.05 were considered significant. All experiments were performed in triplicate.

## SUPPLEMENTARY MATERIALS FIGURES AND TABLE


